# Integrated Experimental Approach, Phytochemistry, and Network Pharmacology to Explore the Potential Mechanisms of *Cinnamomi Ramulus* for Rheumatoid Arthritis

**DOI:** 10.1155/2022/6060677

**Published:** 2022-09-15

**Authors:** Jia Liu, Qing Zhang, Yuanyuan Chen, Lingyu Wang, Ting Tao, Qiang Ren, Xiuping Chen, Yunhui Chen

**Affiliations:** ^1^Chengdu University of Traditional Chinese Medicine, Chengdu 611137, China; ^2^Hospital of Chengdu University of Traditional Chinese Medicine, Chengdu 610072, China; ^3^University of Macau, Macau 999078, China

## Abstract

*Cinnamomi Ramulus* (CR) has been extensively used as a remedy for inflammatory diseases in China. This study adopted an integrative approach of experimental research, phytochemistry, and network pharmacology to investigate its alleviative effects on rheumatoid arthritis (RA) and the underlying potential mechanisms. CR extract (50, 100, and 200 mg/kg) and methotrexate (MTX) significantly ameliorated RA symptoms in the collagen-induced arthritis (CIA) rat model. They also reduced paw volume, arthritis index, proinflammatory cytokines (TNF-*α*, IL-17A, IL-6, and IL-1*β*), and oxidative damage. Sixty-three compounds were systematically identified as the basic components of CR. Fifty-five common genes obtained from compounds and GEO databases were employed to construct the protein-protein interaction (PPI) network. Among them, 20 hub genes were identified via the cytoHubba. Enrichment analysis of the common genes indicated that the TNF signaling pathway and IL-17 signaling pathway might be the potential key pathways. Moreover, molecular docking methods confirmed the high affinity between the top 10 bioactive components of CR and the top 10 targets. In addition, *in vitro* results showed that CR extract (0.2, 0.4, and 0.8 mg/mL) inhibited inflammation and oxidative damage in MH7A cells stimulated by lipopolysaccharide (LPS). In summary, this study adopted multiple approaches to elucidate the protective effect and potential mechanisms of CR on RA, indicating that CR might be a promising herbal candidate for further investigation of RA treatment.

## 1. Introduction

Rheumatoid arthritis (RA) is a progressive inflammatory autoimmune disease that causes severe joint damage, local inflammation, cartilage destruction, and bone erosion. It is associated with multiple genetic and environmental factors, impacts approximately 1% of the population, and is most prevalent among the middle-aged women, imposing a substantial emotional and financial burden on individuals and society [1]. Abnormal activation of fibroblast-like synovial cells (FLS) is the initial event of synovitis and joint injury, leading to bone and cartilage tissue damage, pannus formation, and finally joint destruction [2]. As the disease progresses, patients with RA experience an upsurge of inflammation and oxidative stress, leading to widespread pain from synovitis, progressive histological alterations, and disabling symptoms [3]. Currently, the commonly prescribed drugs for RA include glucocorticoids, nonsteroidal anti-inflammatory drugs (NSAIDs), disease-modifying antirheumatic drugs (DMARDs), and biological therapies [4]. Although these medications are widely prescribed to control the pain, immune responses, and inflammation of RA, their limited efficacy with noticeable side effects are inadequate to address this multifactorial disease. Thus, in order to investigate the pathogenesis of RA and explore valuable natural drugs, bioinformatics approaches should be utilized to identify disease biomarkers and effective targets of natural medicines and clarify their therapeutic effects.

*Cinnamomi Ramulus*, the dried twigs of the aromatic plant *Cinnamomum cassia* (L.) Presl, is an important component of *Guizhi-Shaoyao-Zhimu* decoction (an effective antiarthritic prescription) [5]. According to phytochemistry and pharmacology researches, CR contains a variety of active substances represented by cinnamaldehyde, which have anti-inflammatory, antioxidant, antitumor, antipyretic, and analgesic effects [6]. Modern studies suggested that volatile oil is the main active component of CR, accounting for about 1% of the total medicinal materials [7]. In 2016, Sun et al. found that CR volatile oil alleviates pain and inflammation in mice by inhibiting inflammatory mediator release and iNOS and COX-2 activation [8]. Besides, 80% ethanolic extract of CR exhibited anti-inflammatory and antiarthritic activity by reducing the volume of edema in the CFA-induced chronic arthritic paw of rats [9]. Our previous studies explored its therapeutic value in RA by inhibiting the proliferation, invasion, and migration of fibroblast-like synoviocyte MH7A cells, inducing cell cycle arrest and apoptosis [10]. Certain active compounds in CR may contribute to these biological activities, while their detailed molecular mechanisms remain unclear. With the development of comprehensive bioinformatics analysis, microarray technology provides new insights into identifying key biomarkers for multiple diseases by analyzing data with sophisticated statistical algorithms and investigating overall patterns of gene expression [11]. Network pharmacology is a novel discipline based on system biology, which analyzes the network of biological systems and selects specific signal nodes for a multitarget drug molecule design. In recent years, it has become a pragmatic strategy to decipher the correlations between multicompounds, multitargets, and multipathways of TCM [12].

In this study, the alleviative effect of CR on RA was observed in the collagen-induced arthritis (CIA) rat model. Next, the phytochemical analysis of CR was conducted using ultraperformance liquid chromatography-Q Exactive Orbitrap-mass spectrometry (UPLC-Q Exactive-MS) combined with gas chromatography-mass spectrometry (GC-MS). Then, network pharmacology was employed to systematically decode the potential mechanisms of CR's alleviative actions on RA, and molecular docking was applied to verify the molecular targets. Finally, its potential effects on inhibiting inflammation and oxidative damage were screened *in vitro* based on lipopolysaccharide- (LPS-) induced MH7A cells. This study is aimed at elucidating the therapeutic effect and exploring the potential mechanisms and active ingredients of CR in improving RA, providing useful insight into future drug research and development for RA treatment.

## 2. Materials and Methods

### 2.1. Chemicals and Reagents

*Cinnamomi Ramulus* original material was purchased from the Sichuan New Green Pharmaceutical Technology Development Co., Ltd. (Chengdu, China). Herbal medicine was identified by Prof. Chunjie Wu (School of Pharmacy, Chengdu University of TCM). The bovine type II collagen (CII) was provided by Chondrex Inc. (Chondrex, Seattle, WA, USA). Dimethyl sulfoxide (DMSO), methotrexate (MTX), complete Freund's adjuvant (CFA), and lipopolysaccharide (LPS) were provided by Sigma-Aldrich Co. (St. Louis, MO, USA). The hematoxylin and eosin (H&E) and Safranin O-fast green (SFG) were purchased from Solarbio (Beijing, China). The ELISA assay kits for tumor necrosis factor- (TNF-) *α*, interleukin- (IL-) 1*β*, IL-6, and IL-17A were obtained from Beijing 4A Biotech Co. (Beijing, China). Oxidative stress parameters of superoxide dismutase (SOD), glutathione peroxidase (GSH-Px), catalase (CAT), and malonaldehyde (MDA) were purchased from Suzhou Michy Biomedical Technology Co., Ltd. (Suzhou, China). CCK-8 kits and dihydroethidium (DHE) fluorescent probe were obtained from US Everbright® Inc. (Suzhou, China). The 4′,6-diamidino-2-phenylindole (DAPI) was purchased from BOSTER biological technology company (Wuhan, China). Antibodies against NF-*κ*B p65 and goat-anti-rabbit/rat horseradish-peroxidase-conjugated (HRP) secondary antibodies were purchased from Abcam (Cambridge, MA, USA). High-performance liquid chromatography-grade acetonitrile, methyl alcohol, and formic acid were obtained from Merck KGaA (Merck, Darmstadt, Germany); analytical grade anhydrous diethyl ether, anhydrous sodium sulphate, petroleum ether, ethyl acetate, and n-butyl alcohol were provided by Chengdu Kelong Chemical Co., Ltd. (Chengdu, China).

### 2.2. Preparation of CR Freeze-Dried Powder

The CR freeze-dried powder was prepared as follows. Briefly, the dried plants (200 g) were powdered and soaked with 75% ethanol (1 : 8, *w*/*v*) for 30 min. Reflux extraction was performed 3 times for 1.5 h per time. Each filtrate was combined, and the resulting filtrate mixture was rotationally evaporated at 60°C using a rotary evaporator (EYELA, N-1300V, Tokyo, Japan). The concentrated filtrate was cooled to room temperature, freeze-dried using a lyophilizer (Labconco Co., Kansas, MI, USA) to obtain the dry extract, and stored at 4°C until later use. The yield of the CR extract was 9.85%.

### 2.3. Animals

Specific pathogen-free (SPF) Wistar rats (6-7 weeks old, 200 ± 20 g) were obtained from Chengdu Dossy Experimental Animals Co., Ltd. (Chengdu, China). The animals were acclimated for one week at room temperature (22-24°C) with 50%-65% relative humidity and an alternating 12 h light-dark cycle. All animal experiments were conducted in conformity with the international guidelines for animal experiments and approved by the Animal Care and Use Committee of Chengdu University of Traditional Chinese Medicine.

### 2.4. Establishment of CIA Animal Model and Treatment

Collagen-induced arthritis (CIA) model was prepared according to the description of previous literature [5]. Firstly, bovine type II collagen (2 mg/mL) was emulsified in an equal volume of complete Freund's adjuvant (2 mg/mL). Rats were immunized by subcutaneous injection with 0.1 mL emulsion into the back (left and right sides) and tail base, respectively. The same doses of collagen mixture was performed on day 14 to boost immunization. The normal group was injected with equal volumes of normal saline at the same sites. Rats with CIA on day 21 were randomized into five groups (*n* = 8) based on the volume of hind paw swelling and arthritis score, namely, the CIA model group, CIA+CR (50 mg/kg) group, CIA+CR (100 mg/kg) group, CIA+CR (200 mg/kg) group, and positive control CIA+MTX group (0.2 mg/kg, 3 times/week). CR freeze-dried powder was dissolved in 0.5% CMC-Na solution. Rats in the CR group were given CR freeze-dried powder orally for 24 days, and rats in the normal group and CIA model group were given 0.5% CMC-Na solution in the same volume. Rats in the CR group were given oral administration of CR freeze-dried powder for 24 consecutive days, and the normal group and CIA model group received normal saline simultaneously. Paw volume and arthritis index were measured every three days to evaluate the severity of arthritis. The scoring criteria were as follows: 0 for no erythema or swelling, 1 for slight erythema or swelling of one toe or finger, 2 for erythema and swelling of more than one toe or finger, 3 for erythema and swelling of the ankle or wrist, and 4 for erythema and swelling of all toes or fingers and ankle or wrist [13]. Two hind legs were graded, and a total arthritis score was given for each animal.

### 2.5. Micro-CT Analyses and Histopathological Examination

The hind limb of each rat was harvested after sacrifice and scanned using a PerkinElmer Quantum GX micro-CT system (Norwalk, CT, USA) with the following parameters: X-ray, 90 kV, and 80 *μ*A; field of view (FOV), 72 mm; voxel size, 45-90; scan mode, high resolution; and scan time, 4 min. The 3D reconstruction images were analyzed using the PerkinElmer Analyze software (version 12.0, Norwalk, CT, USA). For histopathological analysis, ankle joints were fixed in 10% formalin after removing the skin and excess tissue. After decalcified in 10% ethylenediaminetetraacetic acid (EDTA) for one month, the samples were embedded in paraffin, sliced into 5 *μ*m sections, stained with H&E, and examined under Nikon TS2 light microscope and high-resolution digital camera system (Nikon TS2, Tokyo, Japan).

### 2.6. Volatile Oil Preparation

In order to explore the main active components in CR, volatile oil was obtained by steam distillation for GC-MS analysis. A total of 200 g of plant material in 0.5 L water were subjected to hydrodistillation for 3 h in a standard apparatus set. The white-yellow or brown oil samples were extracted with anhydrous diethyl ether twice, dried using anhydrous sodium sulphate to remove traces of moisture, and stored in the dark at 4°C until further investigation.

### 2.7. GC-MS Analysis and Compound Identification

The collected essential oil solution was analyzed using a gas chromatography-mass spectrometry (GC-MS) (Agilent 5975C gas chromatography instrument, Agilent Technologies, USA). An HP-5MS capillary column (30 m × 250 *μ*m × 0.25 *μ*m) was employed for the separation. High-purity helium was used as the carrier gas, with a flow rate of 1.0 mL/min. In addition to the injection temperature and interface temperature of 250°C, standard electron impact mass spectrometry source temperature of 230°C and quadrupole temperature of 150°C, the resolution ratio was set as 30 ∶ 1. The full scan monitoring mode was adopted for the mass spectrometry, and the scanning range was m/z 12-550. The column temperature was set at 60°C and programmed to rise at 4°C/min to 200°C (2 min held) and 15°C/min to 290°C (3 min held) kept for 40 min. Upon comparison with the mass spectrometry recorded by the National Institute of Standards and Technology (NIST) mass spectral library, the components contained in CR essential oil were obtained, and the area normalization method was adopted to determine the relative percentage content of each component.

### 2.8. CR Solvent Extraction Preparation

After extracting the volatile oil, the filtrates were concentrated using a vacuum rotary evaporator (Yarong RE 52AA). The obtained concentrate was mixed with water to form a suspension, and the corresponding extraction sections were extracted with petroleum ether, ethyl acetate, and n-butanol successively. Each solvent was extracted 5 times per 200 mL, and the remaining section was the water part. After lyophilization, an appropriate amount of each extracted part was dissolved in methanol and filtered by 0.22 *μ*m microporous membrane. The chemical constituents of each part were qualitatively analyzed by UPLC-Q Exactive-MS.

### 2.9. UPLC-Q Exactive-MS Conditions

Mass spectrum identification was performed using Thermo Scientific Q Exactive Orbitrap HRMS (Thermo Fisher Scientific, Massachusetts, USA) connected to Thermo Scientific Vanquish UPLC (Thermo Fisher Scientific, Massachusetts, USA). Chromatographic separation was achieved on a Thermo ScientificTM AccucoreTM C18 (3 × 100 mm, 2.6 *μ*m) with a flow rate of 0.2 mL/min at 30°C. The mobile phase A was acetonitrile, and the mobile phase B was deionized water (0.1% formic acid). The gradient elution procedures of each part was described in detail: petroleum ether (0-15 min, 40-75% A; 15-30 min,75-85% A; 30-35 min, 85-95% A; 35-40 min, 95-95% A), ethyl acetate (0-15 min, 20-40% A; 15-20 min, 40-80% A; 20-35 min, 80-95% A; 35-40 min, 95-95% A), n-butanol (0-5 min, 10-20% A; 5-15 min, 20-50% A; 15-35 min, 50-95% A; 35-40 min, 95-95% A), and water (0-5 min, 10-30% A; 5-15 min, 30-50% A; 15-25 min, 50-70% A; 25-35 min, 70-95% A; 35-40 min, 95-95% A). After guiding into the electrospray ionization (ESI) source, MS conditions were performed as follows: heath gas flow rate, 35 L/min; spray voltage, 3000 V; capillary temperature, 320°C; aux gas flow rate, 10.00 L/min; and probe heater temperature, 350°C. Full scan spectra were recorded in the mass range of m/z 100-1500. Based on retention time, fragmentation patterns, literature, and the Thermo Scientific™ Compound Discoverer™ software (3.0), the chemical composition was identified in UPLC-Q Exactive-MS positive and negative ion mode.

### 2.10. Network Pharmacology Analysis of CR against RA

#### 2.10.1. Acquisition of RA Targets

In this study, GSE55457 and GSE55235 datasets containing gene expression profiles were downloaded from the Gene Expression Omnibus (GEO) database. Dataset GSE55457, containing synovial tissue samples from 13 RA patients and 10 healthy individuals, was constructed by the Affymetrix Human Genome U133A Array (GPL96 platform). Dataset GSE55235 consisted of 20 samples (10 RA synovial tissue samples and 10 healthy samples) and was based on Affymetrix Human Genome U133A Array (GPL96 platform). To identify the differentially expressed genes (DEGs) between RA and normal samples, GSE55457 and GSE55235 were normalized and visualized by the Limma R package. Based on the threshold of *p* value < 0.05 and |logFC| > 1 judgment, the volcano plot and heat map were obtained through the ggplot2 package and heat map package, respectively. After filtering according to the threshold, these DEGs were collected to form the RA targets library.

#### 2.10.2. Acquisition of CR Targets

We collected the targets of extracted compounds from the Chinese Medicine Systems Pharmacology Database and Analysis Platform (TCMSP), SwissTargetPrediction, PharmMapper online database, and available literature reports [14–17]. After deleting duplicated targets, the Uniprot database was utilized to convert the target names into corresponding gene names to obtain the CR targets library, and then, Cytoscape (3.8.0) software was applied to construct the compound-target network diagram.

#### 2.10.3. Construction of a Protein-Protein Interaction Network

The screened CR and RA targets were imported into the draw Venn diagram for analysis, and overlapping genes were identified as the potential therapeutic targets for CR acting on RA. After the overlapping genes were uploaded to the STRING database, a protein-protein interaction (PPI) network was performed to show interactions between individual targets. The PPI network identified using STRING was further integrated, analyzed, and visualized using the Cytoscape 3.8.0, and hub genes were selected from the PPI networks using the cytoHubba plug-in. Afterwards, a compound-common gene network was constructed by calculating the degrees of each node.

#### 2.10.4. Gene Ontology and Kyoto Encyclopedia of Genes and Genomes Pathway

To comprehensively analyze the biological processes and signaling pathways involved in common genes, the clusterProfiler software package of R (4.0.2) was utilized to perform Gene Ontology (GO) enrichment analysis and Kyoto Encyclopedia of Genes and Genomes (KEGG) pathway analysis. GO biological processes and KEGG pathways with *p* value < 0.05 were considered to be significantly enriched. The top 10 results of GO enrichment and the top 20 results of KEGG pathway enrichment analyses were visualized with bubble plots and column charts by the R software package.

### 2.11. Docking Verification of Compound and Target Molecule

Discovery Studio 4.5 software was used to build the molecular docking model between the top 10 key active ingredients and the top 10 hub genes. We obtained 3D structures of these compounds from ChemDraw software and downloaded “PDB” format files of optimal protein crystal structures for corresponding targets from the RCSB PDB database. Subsequently, ligand and receptor were prepared using Discovery Studio 4.5 software to determine the location of the receptor's active site. Small molecule compounds matching the protein active site were screened by the ligand docking module. The compounds with higher docking scores than the prototype ligand were selected as active molecules.

### 2.12. Cell Culture and Treatment

Human synovial cells MH7A were purchased from the Beina Biological Company (Beijing, China) and cultured in DMEM containing 10% FBS at 37°C in a 5% CO_2_ humidified atmosphere. CCK-8 assay was used to determine the optimal concentration of LPS-induced MH7A cells and the optimal intervention concentration of CR. In brief, MH7A cells (5 × 10^3^) were seeded in 96-well plates and treated with various concentrations of LPS for 6 h [18]. The optimal concentration of LPS-stimulated MH7A cells was treated with CR extract at different doses for 24 h. Then, 10 *μ*L CCK-8 was added to each well and incubated at 37°C for 2 h. The absorbance of each well at 450 nm was measured by an iMARK microplate reader (Bio-Rad, Hercules, CA, USA), and the cell survival rate was calculated.

### 2.13. ELISA Assays of the Proinflammatory Cytokines

Rats were sacrificed, and the serum was collected from the abdominal aorta by centrifugation at 3000 rpm for 15 min and stored at -80°C until assayed. Concentrations of TNF-*α*, IL-1*β*, IL-6, and IL-17A in the serum were measured using ELISA according to the manufacturer's instructions. MH7A cells were treated with LPS (1 *μ*g/mL) for 6 h and then intervened with various doses of CR for 24 h. Then, the concentrations of TNF-*α*, IL-1*β*, IL-6, and IL-17A in MH7A cells were determined using commercial ELISA kits.

### 2.14. Assessment of Oxidative Stress Parameters

All experimental rats were sacrificed, and the serum was obtained by centrifugation at 3000 rpm for 15 min. The serum SOD, CAT, and GSH-Px activities and MDA level were determined by the corresponding assay kit following the manufacturer's protocols. Meanwhile, MH7A cells were treated with LPS (1 *μ*g/mL) for 6 h and then treated with various doses of CR for 24 h. The levels of SOD, CAT, GSH-Px, and MDA in MH7A cells were determined following the manufacturer's protocols.

### 2.15. Determination of Reactive Oxygen Species (ROS)

The DHE fluorescent probe was adopted to detect the level of intracellular reactive oxygen species. In brief, MH7A cells (1 × 10^5^) were incubated in a 6-well plate and treated with LPS and different concentrations of CR. Subsequently, the cells were incubated with DHE (10 *μ*M) for 30 min at 37°C in a dark environment, followed by washing three times with PBS. Cells were collected for intracellular ROS analysis using a FACSCanto II Flow cytometer (BD Company, New York, NY, USA).

### 2.16. Immunofluorescence Assay

MH7A cells were seeded into a confocal laser dish and treated with LPS and different concentrations of CR. At the end of the intervention, the cells were fixed with 4% paraformaldehyde for 20 min and then permeated with 0.1% Triton X-100 in PBS for 1 h at room temperature. The cells were incubated with NF-*κ*B p65 antibody (diluted 1 : 200) overnight at 4°C. Anti-rabbit IgG (H+L) Alexa Fluor® was incubated at room temperature for 1 h in the dark, and the nuclei were visualized using DAPI staining. After washing with PBS for three times, the fluorescence intensity was observed using a confocal laser microscope (Leica, SP8 SR, Wetzlar, Germany).

### 2.17. Statistical Analysis

Data were expressed as mean ± standard deviation. Differences between multiple groups were assessed using one-way analysis of variance. *p* values < 0.05 were deemed statistically significant. Analysis and graphing were completed utilizing GraphPad Prism 8.0 software (San Diego, CA, USA).

## 3. Results

### 3.1. CR Alleviated the Severity of RA in CIA Rats

As shown in Figure 1(a), the CIA rat model was established to validate the efficacy of CR against RA. Photographs of paw edema showed that joint swelling in CIA rats was significantly reduced after 24 days of MTX and CR treatment (Figure 1(b)). The arthritis index in CIA rats peaked on day 9 after administration (day 30 after primary immunization) compared with the normal control group. After MTX and CR treatment, arthritic symptoms and arthritic scores of CIA rats were significantly improved (Figures 1(c) and 1(d)). As shown in Figure 1(e), the levels of inflammatory cytokines (TNF-*α*, IL-1*β*, IL-6, and IL-17A) were significantly higher in the model group than in the normal group. The results of the CR group and MTX group were consistent, and the effects of different CR concentrations on TNF-*α*, IL-1*β*, IL-6, and IL-17A levels were dose-dependent. As displayed in Figure 1(f), CIA rats developed oxidative stress with a decreased antioxidant enzyme activity (SOD, CAT, and GSH-Px) and an increased serum MDA level compared to the normal group. However, CR and MTX treatments were observed to significantly reduce oxidative damage. As expected, intervention of CR at different doses (50, 100, and 200 mg/kg) significantly reduced the serum level of MDA and elevated the activity of antioxidant enzyme.

### 3.2. CR Inhibited Ankle and Cartilage Damage in CIA Rats

The results of H&E and Safranin O staining demonstrated that the ankle joint and synovial tissue in the normal group were intact without damage. On the contrary, synovial cell proliferation and inflammatory cell infiltration were noted in the model group. CR (50, 100, and 200 mg/kg) and MTX treatment all reduced synovial hyperplasia, synovial inflammation, and cartilage erosion in CIA rats. Micro-CT imaging revealed that normal rats had smooth articular surface, clear and complete articular structure, normal bone and articular space, and absence of soft tissue swelling. CIA rats showed joint surface fusion, joint space narrowing, severe structural erosion, and destructive bone resorption and dissolution. CR and MTX intervention reduced soft tissue swelling and bone destruction, as well as deterioration of articular surface structure and space clarity (Figure 2(a)). The quantitative analysis for synovitis and cartilage damage is shown in Figures 2(b) and 2(c).

### 3.3. Analysis of the Constituents of Volatile Oil Obtained from CR

A total of 28 volatile compounds were identified utilizing the NIST mass spectral library and literature data [19–21] (Figure 3(a)). The retention time, formula, molecular weight, and area percentage of benzaldehyde (1), 4-hydroxybenzaldehyde (2), acetophenone (3), benzenepropanal (4), linderol (5), (-)-alpha-terpineol (6), *cis*-cinnamaldehyde (7), 3-phenylpropanol (8), 2-methoxybenzaldehyde (9), cinnamaldehyde (10), alpha-copaene (11), beta-caryophyllene (12), coumarin (13), cinnamyl acetate (14), gamma-muurolene (15), alpha-curcumene (16), alpha-muurolene (17), beta-bisabolene (18), trans-calamenene (19), 2-methoxycinnamaldehyde (20), alpha-calacorene (21), spathulenol (22), cedrol (23), tetradecanal (24), tau-cadinol (25), alpha-cadinol (26), cadalene (27), and alpha-bisabolol (28) are shown in Table 1. The structures of these compounds are presented in Figure 3(b).

### 3.4. Identification and Analysis of Active Constituents in CR Extract

Total ion chromatograms of each part in positive and negative ion modes are presented in Figures 4(a)–4(d). A total of 35 compounds were preliminarily isolated and identified from CR extract, including azelaic acid (29), syringaldehyde (30), coniferyl aldehyde (31), caryophyllene oxide (32), benzyl cinnamate (33), oleoyl ethanolamide (34), oleamide (35), stearoyl ethanolamide (36), stearamide (37), benzoic acid (38), catechin (39), 4-methoxybenzaldehyde (40), caffeic acid (41), 4-methoxycinnamaldehyde (42), p-coumaric acid (43), quercetin (44), taxifolin (45), ferulic acid (46), kaempferol (47), cinnamic acid (48), methyl eugenol (49), methyl cinnamate (50), ethyl 4-methoxycinnamate (51), 4-methoxycinnamic acid (52), 2-hydroxycinnamic acid (53), 3,4-dimethoxycinnamic acid (54), 2,3-dihydroxybenzoic acid (55), syringic acid (56), 2,4-dihydroxybenzoic acid (57), sebacic acid (58), 2-methoxybenzoic acid (59), 2-methoxycinnamic acid (60), isoquercetin (61), kaempferol-3-O-glucoside (62), and quercitrin (63) [22–42]. The retention time, formula, molecular weight, error value, fragment ion, and other details of 35 compounds are shown in Table 2, and the structures of these compounds are displayed in Figure 4(e).

### 3.5. Results of Network Pharmacology Analysis

#### 3.5.1. Prediction of Related Targets of RA

After standardized processing of the two datasets downloaded from the GEO database, 419 DEGs were obtained from the RA synovial tissues and normal controls, including 183 upregulated genes (red dots) and 236 downregulated genes (green dots). Volcano map and heat map analysis of the DEGs were performed by R software (Figures 5(a) and 5(b)).

#### 3.5.2. Prediction of Anti-RA Targets of CR

We obtained targets for 63 compounds from TCMSP, PharmMapper, and SwissTargetPrediction databases, and a total of 559 unduplicated targets were collected. A compound-target network was constructed based on the interaction relationship between these 63 compounds and their corresponding targets (Figure 5(c)). The network consists of 622 nodes (63 compounds and 559 targets) and 2075 edges. Red circular nodes represent compounds, blue circular nodes symbolize targets, green circular nodes represent common targets, and edges symbolize interactions between compounds and targets. The 559 active compound targets and the 419 disease targets were used to draw a Venn diagram, and 55 common targets were obtained (Figure 5(d)).

#### 3.5.3. Compound-Common Gene Network

The PPI network was obtained by importing 55 common targets into STRING and removing five disconnected points. The downloaded TSV data were imported into Cytoscape 3.8.0 to visualize the protein interaction network, with darker node colors representing larger degree values (Figure 6(a)). The 20 hub targets were calculated by the cytoHubba plug-in, and the ranks were represented by color changes from red to yellow (Figure 6(b)). After removing 12 compounds without related targets, 51 active candidate compounds were obtained. Cytoscape 3.8.0 was utilized to construct a network diagram of 51 compounds and 55 common gene targets, as shown in Figure 6(c), consisting of 106 nodes and 244 edges. The results showed that cinnamaldehyde (10), caffeic acid (41), benzyl cinnamate (33), cinnamyl acetate (14), 4-methoxy-cinnamaldehyde (42), 2-methoxy-cinnamaldehyde (20), quercetin (44), kaempferol (47), 3, 4-dimethoxy-4-methoxy-cinnamic acid (52), cinnamic acid (54), ethyl 4-methoxycinnamate (51), 4-methoxy-benzaldehyde (40), 2-methoxybenzaldehyde (9), and coniferyl aldehyde (31) might be candidate bioactive substances for the treatment of RA.

#### 3.5.4. GO and KEGG Pathway Enrichment Analyses

We performed GO and KEGG pathway enrichment analyses to further elucidate the biological functions of 55 common genes systematically. As shown in Figure 6(d), the top 10 terms in the BPs, CCs, and MFs were selected. The enrichment of BPs involved the regulation of cytosolic calcium ion concentration, cell chemotaxis, regulation of inflammatory response, and cellular calcium ion homeostasis. Enrichment to CCs mainly included membrane raft, membrane microdomain, and membrane region. The MFs most enriched in protein serine/threonine kinase activity, metallopeptidase activity, and metalloendopeptidase activity. Additionally, the KEGG pathways were most enriched in apoptosis and inflammatory-associated pathways, such as the TNF signaling pathway, osteoclast differentiation, IL-17 signaling pathway, apoptosis, Th17 cell differentiation, Th1 and Th2 cell differentiation, rheumatoid arthritis, and NF-kappa B signaling pathway. The top 20 pathways are shown in Figure 6(e).

### 3.6. Molecular Docking Verification

We searched the 3D structure of these 10 hub genes in the PDB database: IL6 (PDB: 4CNI), MAPK8 (PDB: 4HYS), PTGS2 (PDB: 5KIR), JUN (PDB: 2NO3), CCL5 (PDB: 5UIW), STAT1 (PDB: 6HHO), FOS (PDB: 6W3E), IL1R1 (PDB: 4GAF), SOCS3 (PDB: 6C7Y), and MAPK14 (PDB: 6SFO). The higher the molecular docking score, the better the receptor-ligand binding ability. According to Figure 7, the optimal docking results of the 10 hub genes and the top 10 bioactive compounds were presented in 3D topological structures of the drug-target binding model. Notably, these compounds were closely bound to the receptors through hydrogen bonds, hydrophobic interaction of amino acids, and *π*-conjugated effects. The above results indicated that the interaction between these core targets and core components was the biological basis for the multitarget action of CR against RA.

### 3.7. CR Ameliorated LPS-Induced Inflammatory Injury in MH7A Cells

MH7A cells were treated with different doses of LPS for 6 h to establish the LPS-induced inflammatory injury model. As shown in Figure 8(a), 1 *μ*g/mL of LPS increased the viability of MH7A cells compared to the untreated control group, while LPS-induced survival decreased from 4 *μ*g/mL. Given the effect of LPS on enhancing the viability of MH7A cells, 1 *μ*g/mL LPS was selected as the stimulation condition for subsequent experiments. LPS-induced MH7A cells were treated with different doses of CR to detect cytotoxicity. Data in Figure 8(b) showed that 0.2 mg/mL CR began to decrease the viability of MH7A cells compared with the LPS group. Thus, 0.2, 0.4, and 0.8 mg/mL were selected as a CR-intervention condition for follow-up experiments. Since inflammation is a major contributor to LPS damage, the release of proinflammatory cytokines was also measured in this study. ELISA assay showed that CR significantly decreased the LPS-induced release of four proinflammatory cytokines (Figure 8(c)). NF-*κ*B plays a crucial role in modulating synovial inflammation and joint destruction. Immunofluorescence results were shown in Figure 8(d), indicating that the activated NF-*κ*B P65 in MH7A cells was significantly translocated into the nucleus after LPS treatment. However, this translocation effect was restrained by CR.

### 3.8. CR Ameliorated LPS-Induced Oxidative Stress in MH7A Cells

The effect of CR treatment on ROS overproduction in LPS-stimulated MH7A cells was determined by the DHE probe. The results showed that ROS accumulation in 1 *μ*g/mL LPS-induced cells increased dramatically compared with normal cells. However, CR treatment significantly reduced the intracellular ROS production in LPS-induced MH7A cells (Figure 9(a)). In addition, the antioxidant activity of CR was evaluated by determining the contents of antioxidant enzymes SOD, CAT, GSH-Px, and lipid peroxidation product MDA in LPS-induced MH7A cells. As shown in Figure 9(b), the MDA content of MH7A cells was significantly increased after LPS treatment, while activities of SOD, CAT, and GSH-Px were decreased. Nevertheless, the level of MDA was significantly downregulated and the activities of SOD, CAT, and GSH-Px were upregulated after CR treatment, indicating CR at different doses exerted therapeutic effects. These results suggested that CR could balance the LPS-induced oxidative stress in MH7A cells, which might be associated with the increased ROS scavenging enzyme activity.

## 4. Discussion

*Cinnamomi Ramulus* is a commonly prescribed Chinese medicine for arthritis treatment. There are many effective antiarthritis prescriptions containing CR in the Chinese Pharmacopoeia, and some studies on the anti-inflammatory and antiarthritic effects of CR in animal models of RA have been published. Notably, in addition to CR volatile oil and its extracts significantly alleviating inflammation and pain in CFA-induced chronic arthritis rats, active components such as cinnamaldehyde in CR volatile oil could also reduce RA symptoms by ameliorating oxidative stress and the release of inflammatory factors [14, 15]. However, due to the complex chemical composition of CR, its potential active components and the exact pharmacological mechanism for the treatment of RA remain difficult to elucidate. In our study, a comprehensive investigation approach integrating the CIA rat model, GC-MS, UPLC-Q Exactive-MS analysis, and bioinformatics were adopted to reveal the material basis and molecular mechanism of CR for RA treatment, and corresponding *in vitro* data were provided for verification.

A CIA rat model with similar clinical symptoms and pathological changes to RA was used for the *in vivo* exploration. Compared with the normal group, CIA rats showed obvious arthritis symptoms such as joint swelling, increased paw volume, and arthritic index. Since the initial phase of RA involves an imbalance of proinflammatory and anti-inflammatory cytokine activities, increasing proinflammatory cytokines such as TNF-*α*, IL-6, and IL-17 could stimulate inflammation and degradation of bone and cartilage [43]. Therefore, analysis of the expression of inflammatory cytokines has been deemed an important index to study the occurrence of RA. In this study, ELISA results showed that serum levels of inflammatory cytokines TNF-*α*, IL-17A, IL-1*β*, and IL-6 in CIA rats were higher than in the normal group, while MTX and CR extract significantly reversed these changes. In addition to inflammatory factors, the total ROS in peripheral blood and synovial tissue of RA patients were also significantly increased. After ROS inhibitor treatment, the expression of inflammatory cytokines in RA-FLS was distinctly inhibited [44]. As part of the endogenous antioxidant system, SOD, CAT, and GSH-Px protect tissues from oxidative damage by scavenging free radical superoxides. MDA is a decomposition product of lipid hydroperoxides and is correlated with the increased oxidative stress activity in inflammatory sites [45]. Our study demonstrated that CR attenuated the lipid peroxidation, enhanced the activity of antioxidant defense enzymes, and inhibited the oxidative stress state in RA rats. The H&E and safranin O-fast green staining results revealed that the cartilage tissue structure in the model group was significantly changed with hyperplastic and disordered synovial cells and infiltrating inflammatory cells, while CR extract could improve these pathological changes. Micro-CT scanning imaging results demonstrated that normal rats had obvious articular space, clear articular structure, and no bone erosion or hyperplasia changes, while CIA rats presented bone erosion-like changes, coarse articular surface, and notably narrowed joint space. After CR treatment, only slight erosive changes and joint space narrowing were observed in CIA rats.

Furthermore, 63 compounds were identified from the volatile oil and extract of CR, among which cinnamaldehyde, caffeic acid, benzyl cinnamate, cinnamyl acetate, 4-methoxy-cinnamaldehyde, and quercetin were closely correlated with anti-RA bioactivity. Cinnamaldehyde effectively ameliorated oxidative stress and inflammation in RA rats by activating enzymatic antioxidants and inhibiting the release of pro-inflammatory factors (TNF-*α*, IL-6, and IL-10) [14]. Caffeic acid not only mitigated adjuvant-induced paw edema and inflammatory cell infiltration in arthritic rats but also lowered the paw expression of NF-*κ*B, chitinase-3-like protein-1, and angiogenesis [46]. Quercetin provided better protection against arthritis than MTX in terms of body weight, edema, joint damage, and cytokine production in mice [47]. Multiple compounds of CR acted on multiple targets at the same time, indicating that the anti-RA effect of CR was realized through the synergistic interaction of its compounds. IL6, MAPK8, PTGS2, JUN, and CCL5 were the core target proteins of CR for the treatment of RA. IL-6 is a highly expressed proinflammatory cytokine in the rheumatoid synovium, causing inflammation, pannus formation, and cartilage destruction. As an established target for the treatment of RA, its receptor antagonist tocilizumab has been widely accepted in the market [48]. The mitogen-activated protein kinase (MAPKs) signaling cascade is involved in the inflammation and tissue destruction of RA [49]. C-Jun N-terminal kinase (JNK) is highly activated in RA fibroblast-like synovial cells and synovium, which participated in cellular inflammation and cartilage degradation [50]. Selective cyclooxygenase-2 (COX-2) inhibitors (such as celecoxib) are commonly utilized to treat RA due to their significant anti-inflammatory, analgesic, and antipyretic activities [51]. Chemokine (C-C motif) ligand 5 (CCL5) regulates the immunopathological mechanism of RA joint inflammation and also increases MMP expression to induce collagen degradation [52]. The main compounds in CR binded well to these core proteins, which was further confirmed by molecular docking. These results provide supporting evidence that cinnamaldehyde, caffeic acid, benzyl cinnamate, cinnamyl acetate, 4-methoxy-cinnamaldehyde, and quercetin may be the main active compounds of CR in the treatment of RA, as they affect most of the targets associated with RA.

The actions of CR on RA are primarily based on effective pathophysiological mechanisms. According to the functional enrichment analysis results, CR interferes with the occurrence and development of RA mainly through the TNF signaling pathway, osteoclast differentiation, IL-17 signaling pathway, apoptosis, Th17 cell differentiation, and NF-kappa B signaling pathway. TNF is a pleiotropic cytokine widely involved in multiple aspects of RA modulation, and anti-TNF biological therapy has been deemed a second-line treatment for RA after methotrexate [53]. High levels of IL-17 produced by Th17 cells in RA promote osteoclast formation, bone resorption, marginal erosions, and release of other proinflammatory cytokines [54]. NF-*κ*B is an important regulator of inflammatory response and immune stability, controlling normal development and the pathological destruction of cartilage. Meanwhile, NF-*κ*B pathway is the major upstream signaling pathway controlling the production of TNF-*α*, IL-1*β*, IL-6, and IL-17A [55]. In the current study, MH7A cells were treated with LPS to establish the RA cell model. LPS stimulated MH7A cells to generate proinflammatory cytokines, such as TNF-*α*, IL-1*β*, IL-6, and IL-17A, and increased NF-*κ*B P65 nuclear translocation. However, cells treated with CR significantly attenuated LPS-triggered inflammatory damage. RA symptoms are also attributed to oxidative imbalance, with ROS resulting in altered chondrocyte metabolic function, which subsequently leads to impaired extracellular matrix synthesis and activation of inflammatory-related events [56]. Consequently, in addition to the inflammatory pathway, we further observed that CR treatment could upregulate the activities of SOD, CAT, and GSH-Px and downregulate the levels of ROS and MDA in a concentration-dependent manner, indicating that CR maintained ROS homeostasis in MH7A cells. Therefore, these results suggested that inhibition of ROS-NF-*κ*B-related inflammation and oxidative damage is an effective pathway for CR to relieve RA.

## 5. Conclusion

In summary, the present study revealed the protective effect of CR on experimental RA cartilage destruction and inflammation. Specifically, its effects against RA were mediated via improving synovial hyperplasia and inflammation, reducing ROS-mediated lipid peroxidation, and enhancing antioxidant defense mechanisms. Hopefully, this study may also provide useful insight for screening and investigating the complex pharmacodynamic components and mechanisms of natural medicine.

## Figures and Tables

**Figure 1:** CR attenuated CIA-induced RA in rats. (a) The experimental procedure was illustrated. (b) Representative photographic images of rats in different treatment groups. (c) Effects of CR extract on paw volume of CIA rats. (d) Effects of CR extract on arthritis index of CIA rats. (e) Effects of CR extract on serum levels of pro-inflammatory cytokines (TNF-*α*, IL-17A, IL-6, and IL-1*β*). (f) Effects of CR extract on serum SOD, CAT, GSH-Px, and MDA levels. Data are expressed as mean ± SD; ^∗^*p* < 0.05, ^∗∗^*p* < 0.01 vs. the model group.

**Figure 2:** Effects of CR on histopathological changes and joint destruction of CIA rats. (a) Representative H&E staining and Safranin O staining of ankle joint sections, and representative images of the micro-CT determination. The quantitative results for (b) synovitis and (c) cartilage damage. Data are expressed as mean ± SD; ^∗^*p* < 0.05, ^∗∗^*p* < 0.01 vs. the model group.

**Figure 3:** (a) The total ion chromatograms of volatile oil from *Cinnamomi Ramulus.* (b) Compounds in volatile oil from *Cinnamomi Ramulus*.

**Figure 4:** The total ion chromatograms of different fractions of *Cinnamomi Ramulus*: (a) petroleum ether fraction, (b) ethyl acetate fraction, (c) n-butanol fraction and (d) water fraction. (e) Compounds in different fractions of *Cinnamomi Ramulus*.

**Figure 5:** Prediction of anti-RA targets of CR. (a) Volcano map of DEGs in the GSE55235 and GSE55457 microarray datasets, with logFC on the vertical axis and log10 (*p* value) on the horizontal axis. (b) Heat map of DEGs in the GSE55235 and GSE55457 microarray datasets, with the vertical axis representing samples and the horizontal axis representing differentially expressed genes. (c) Compound-target network. The red circular node, blue ellipse nodes, and green ellipse nodes represented the compounds, targets, and overlapping genes, respectively. (d) Common genes between DEGs and compound targets.

**Figure 6:** GO and KEGG enrichment analysis results. (a) PPI networks for common genes. (b) The top 20 hub genes of the common genes. (c) Active compound-common gene network. (d) The top 10 items with significant enrichment in BP, CC, and MF of GO analysis. The *y*-axis represents the enrichment count of target genes, and the *x*-axis represents the GO category of target genes. (e) The KEGG analysis diagram including the top 20 significant enrichment pathways. The *y*-axis represents the enrichment pathways, and the *x*-axis represents the enrichment score.

**Figure 7:** Molecular docking results of the 10 hub genes and the top 10 bioactive compounds: (a) IL6 and 44, (b) MAPK8 and 47, (c) PTGS2 and 33, (d) JUN and 47, (e) CCL5 and 10, (f) STAT1 and 42, (g) FOS and 54, (h) IL1R1 and 51, (i) SOCS3 and 14, and (j) MAPK14 and 41.

**Figure 8:** CR inhibited inflammation in LPS-induced MH7A cells. (a) The cell viability of MH7A cells treated with various doses of LPS for 6 h. (b) The cell viability of LPS-induced MH7A cells treated with different concentrations of CR for 24 h. (c) Effects of CR extract on the levels of proinflammatory cytokines (TNF-*α*, IL-17A, IL-6, and IL-1*β*) in LPS-induced MH7A cells. (d) Effect of CR on LPS-induced nuclear translocation of NF-*κ*B p65. Data are expressed as mean ± SD; ^∗^*p* < 0.05, ^∗∗^*p* < 0.01 vs. the model group.

**Figure 9:** CR maintained redox balance in LPS-induced MH7A cells. (a) Effects of CR extract on ROS levels in LPS-stimulated MH7A cells. (b) Effects of CR extract on SOD, CAT, GSH-Px, and MDA levels in LPS-induced MH7A cells. Data are expressed as mean ± SD; ^∗^*p* < 0.05, ^∗∗^*p* < 0.01 vs. the model group.

**Table 1:** Compounds identified in volatile oil from CR.

Peak no.	RT (min)	Compound	Formula	Molecular weight	Relative amount (%)
1.	5.705	Benzaldehyde	C_7_H_6_O	106.12	0.74
2.	7.947	4-Hydroxybenzaldehyde	C_7_H_6_O_2_	122.12	0.1
3.	8.64	Acetophenone	C_8_H_8_O	120.15	0.97
4.	11.722	Benzenepropanal	C_9_H_10_O	134.17	0.74
5.	11.918	Linderol	C_10_H_18_O	154.25	0.19
6.	12.696	Alpha-terpineol	C_10_H_18_O	154.25	0.08
7.	13.621	*cis*-Cinnamaldehyde	C_9_H_8_O	132.16	1.20
8.	14.252	3-Phenylpropanol	C_9_H_12_O	136.19	0.22
9.	14.393	2-Methoxybenzaldehyde	C_8_H_8_O_2_	136.15	0.32
10.	15.919	*trans*-Cinnamaldehyde	C_9_H_8_O	132.16	88.30
11.	18.719	Alpha-copaene	C_15_H_24_	204.35	0.22
12.	20.116	Beta-baryophyllene	C_15_H_24_	204.35	0.09
13.	20.729	Coumarin	C_9_H_6_O_2_	146.14	0.21
14.	20.962	Cinnamyl acetate	C_11_H_12_O_2_	176.21	0.28
15.	21.899	Gamma-muurolene	C_15_H_24_	204.35	0.11
16.	22.095	Alpha-curcumene	C_15_H_22_	202.33	0.2
17.	22.628	Alpha-muurolene	C_15_H_24_	204.35	0.1
18.	22.867	Beta-bisabolene	C_15_H_24_	204.35	0.16
19.	23.327	*trans*-Calamenene	C_15_H_22_	202.33	0.19
20.	23.639	2-Methoxycinnamaldehyde	C_10_H_10_O_2_	162.18	2.88
21.	23.939	Alpha-calacorene	C_15_H_20_	200.32	0.14
22.	25.018	Spathulenol	C_15_H_24_O	220.35	0.45
23.	25.729	Cedrol	C_15_H_26_O	222.37	0.08
24.	25.912	Tetradecanal	C_14_H_28_O	212.37	0.12
25.	26.844	Tau-cadinol	C_15_H_26_O	222.37	0.23
26.	27.218	Alpha-cadinol	C_15_H_26_O	222.37	0.13
27.	27.781	Cadalene	C_15_H_18_	198.3	0.12
28.	28.075	Alpha-bisabolol	C_15_H_26_O	222.37	0.25

**Table 2:** Compounds identified in the CR by UPLC-QE-MS/MS.

Peak no.	RT (min)	Formula	Molecular weight	ESI-MS	Error (ppm)	Fragment ions (m/z)	Name	Ref
29	1.94	C_9_H_16_O_4_	188.10469	187.09741[M-H]^−^	-0.9	169, 125, 97	Azelaic acid	22
30	2.509	C_9_H_10_O_4_	182.05843	183.06576[M+H]^+^	2.85	168, 155, 140, 123, 95	Syringaldehyde	23
31	2.98	C_10_H_10_O_3_	178.06265	179.06978[M+H]^+^	-1.93	164, 161, 147, 133, 119, 105, 55	Coniferyl aldehyde	24
32	6.763	C_15_H_24_O	220.18333	221.19066[M+H]^+^	2.81	207, 175, 161, 147, 133, 121, 109, 95, 81, 69, 55	Caryophyllene oxide	25
33	9.261	C_16_H_14_O_2_	238.09984	239.10710[M+H]^+^	1.93	192, 131, 91	Benzyl cinnamate	26
34	18.823	C_20_H_39_NO_2_	325.29875	326.30603[M+H]^+^	2.07	308, 62	Oleoyl ethanolamide	27
35	27.451	C_18_H_35_NO	281.27245	282.27982[M+H]^+^	2.07	97, 83, 55	Oleamide	28
36	30.611	C_20_H_41_NO_2_	327.31456	328.32178[M+H]^+^	2.54	311, 62	Stearoyl ethanolamide	29
37	34.293	C_18_H_37_NO	283.2883	284.29556[M+H]^+^	2.7	266, 88, 57	Stearamide	30
38	1.981	C_7_H_6_O_2_	122.03708	121.04431[M-H]^−^	2.44	93, 65	Benzoic acid	31
39	1.999	C_15_H_14_O_6_	290.07902	289.08643[M-H]^−^	-0.07	245, 203, 151, 125, 109, 97	Catechin	22
40	2.813	C_8_H_8_O_2_	136.05254	137.05983[M+H]^+^	0.84	122, 109, 94	4-Methoxybenzaldehyde	23
41	2.861	C_9_H_8_O_4_	180.04176	179.03433[M-H]^−^	-2.76	135, 107	Caffeic acid	22
42	2.947	C_10_H_10_O_2_	162.06806	163.07544[M+H]^+^	0.05	145, 135, 121, 105, 79, 55	4-Methoxycinnamaldehyde	26
43	4.396	C_9_H_8_O_3_	164.04719	163.03949[M-H]-	-0.93	119, 93	p-Coumaric acid	22
44	4.584	C_15_H_10_O_7_	302.0428	303.05014[M+H]^+^	0.5	257, 229, 201, 165, 153, 137	Quercetin	32
45	5.018	C_15_H_12_O_7_	304.05854	303.05130[M-H]^−^	-3.62	285, 217, 151, 125, 109	Taxifolin	22
46	5.661	C_10_H_10_O_4_	194.0578	193.05026[M-H]^−^	-0.59	161, 151, 134	Ferulic acid	33
47	5.863	C_15_H_10_O_6_	286.04805	287.05533[M+H]^+^	1.1	165, 153	Kaempferol	32
48	6.15	C_9_H_8_O_2_	148.05288	149.04446[M+H]^+^	-4.55	131, 123, 103	Cinnamic acid	26
49	8.789	C_11_H_14_O_2_	178.0629	179.07045[M+H]^+^	-0.54	103, 91	Methyl eugenol	34
50	10.21	C_10_H_10_O_2_	162.06814	163.07553[M+H]^+^	0.4	131, 103, 95	Methyl cinnamate	35
51	11.111	C_12_H_14_O_3_	206.09453	207.10184[M+H]^+^	1.13	161, 134, 133	Ethyl 4-methoxycinnamate	36
52	12.743	C_10_H_10_O_3_	178.06343	179.07039[M+H]^+^	1.34	133, 117, 105	4-Methoxycinnamic acid	35
53	18.67	C_9_H_8_O_3_	164.04758	165.05475[M+H]^+^	1.43	147, 123, 103, 91	2-Hydroxycinnamic acid	26
54	2.013	C_11_H_12_O_4_	208.0738	209.08141[M+H]+	0.92	191, 163, 91	3,4-Dimethoxycinnamic acid	37
55	3.699	C_7_H_6_O_4_	154.0259	153.0186[M-H]-	-4.57	153, 109	2,3-Dihydroxybenzoic acid	38
56	5.75	C_9_H_10_O_5_	198.0534	197.06065[M-H]-	2.8	182, 167, 153, 139, 123	Syringic acid	22
57	7.366	C_7_H_6_O_4_	154.0259	153.01859[M-H]-	-4.85	153, 109	2,4-Dihydroxybenzoic acid	38
58	9.367	C_10_H_18_O_4_	202.1203	201.12743[M-H]-	-1.04	183, 139	Sebacic acid	39
59	11.23	C_8_H_8_O_3_	152.0477	153.05493[M+H]+	2.09	135, 92, 77	2-Methoxybenzoic acid	40
60	11.561	C_10_H_10_O_3_	178.063	179.07036[M+H]+	-0.01	161, 131, 103, 77	2-Methoxycinnamic acid	41
61	8.225	C_21_H_20_O_12_	464.0958	463.08865[M-H]-	0.66	317, 287, 259, 151, 125, 109	Isoquercetin	22
62	9.335	C_2_1H_20_O_11_	448.101	447.09409[M-H]-	0.97	285, 255, 227	Kaempferol-3-O-glucoside	31
63	9.496	C_21_H_20_O_11_	448.101	447.09372[M-H]-	0.97	301, 300, 255, 179	Quercitrin	42

## Data Availability

The datasets generated for this study are available.

## Abbreviations

BP: Biological process
CC: Cellular component
CIA: Type II collagen-induce arthritis
CR: *Cinnamomi Ramulus*
CXCL8: C-X-C motif chemokine ligand 8
DAVID: Database for Annotation, Visualization and Integrated Discovery
DMARDs: Disease-modifying antirheumatic drugs
EDTA: Ethylenediaminetetraacetic acid
ELISA: Enzyme-linked immunosorbent assays
ESI: Electrospray ionization
GC-MS: Gas chromatography-mass spectrometry
GEO: Gene Expression Ominibus
GO: Gene Ontology
H&E: Hematoxylin and eosin
IL: Interleukin
KEGG: Kyoto Encyclopedia of Genes and Genomes
MAPK: Mitogen-activated protein kinase
MF: Molecular function
MMP: Matrix metalloproteinases
MTX: Methotrexate
NIST: National Institute of Standards and Technology
NSAIDs: Nonsteroidal anti-inflammatory drugs
PDB: Protein Data Bank
PPI: Protein-protein interaction
RA: Rheumatoid arthritis
STRING: Search Tool for the Retrieval of Interacting Genes/Proteins
TCM: Traditional Chinese medicine
TCMSP: Traditional Chinese medicine systems pharmacology database and analysis platform
TNF: Tumor necrosis factor
UPLC-Q Exactive-MS: Ultraperformance liquid chromatography-Q Exactive Orbitrap-mass spectrometry.
